The article "Automatic Segmentation of MRI of Brain Tumor Using Deep Convolutional Network" was retracted in 2023. Reasons: signs of a paper mill; compromised peer review; unreliable results or conclusions.

# Automatic Segmentation of MRI of Brain Tumor Using Deep Convolutional Network

**DOI:** 10.1155/2022/4247631

**Published:** 2022-06-15

**Authors:** Runwei Zhou, Shijun Hu, Baoxiang Ma, Bangcheng Ma

**Affiliations:** Department of Radiology, Wenzhou Seventh People's Hospital, Ouhai District, Wenzhou City, Zhejiang Province 325006, China

## Abstract

Computer-aided diagnosis and treatment of multimodal magnetic resonance imaging (MRI) brain tumor image segmentation has always been a hot and significant topic in the field of medical image processing. Multimodal MRI brain tumor image segmentation utilizes the characteristics of each modal in the MRI image to segment the entire tumor and tumor core area and enhanced them from normal brain tissues. However, the grayscale similarity between brain tissues in various MRI images is very immense making it difficult to deal with the segmentation of multimodal MRI brain tumor images through traditional algorithms. Therefore, we employ the deep learning method as a tool to make full use of the complementary feature information between the multimodalities and instigate the following research: (i) build a network model suitable for brain tumor segmentation tasks based on the fully convolutional neural network framework and (ii) adopting an end-to-end training method, using two-dimensional slices of MRI images as network input data. The problem of unbalanced categories in various brain tumor image data is overcome by introducing the Dice loss function into the network to calculate the network training loss; at the same time, parallel Dice loss is proposed to further improve the substructure segmentation effect. We proposed a cascaded network model based on a fully convolutional neural network to improve the tumor core area and enhance the segmentation accuracy of the tumor area and achieve good prediction results for the substructure segmentation on the BraTS 2017 data set.

## 1. Introduction

The tumor is a lump of tissue caused by the proliferation of certain tissue cells in the body under the influence of tumor-causing factors. It is a malignant disease endangering human health. Brain tumors refer to uncontrolled cell growth in the cranial cavity which can be categorized as primary and secondary on basis of origin. Primary tumors can be subcategorized as intramedullary tumors and extramedullary tumors. The intramedullary area mainly includes gliomas which are most likely derived from the neuroepithelium, which is relatively a common primary tumor. The incidence of brain tumors constitutes 1.4% of systemic tumors, and the occurrence of glioma is about 40% to 50% of intracranial tumors. Glioma is a very fatal disease having an average of 2.4% mortality rate among 20-50-year-old patients [1, 2]. Based on diagnosis, tumors can be classified as benign or malignant. Benign tumors are relatively slow to grow and can have a longer survival time; while malignant tumors grow faster in general, patients can only survive for two years or less. Early detection of the lesion area in the clinic and targeted treatment of the affected area is one of the effective ways to minimize the risk of brain tumors.

The region-based segmentation method is a classic image processing method. Its processing is mainly based on the similar features of the pixels in the region like texture characteristics and image gray value. Region-based segmentation methods generally utilized fuzzy *C*-means, *K*-means clustering, threshold segmentation, Gaussian mixture model, morphological watershed segmentation, region growth, Markov-based random field, and other methods. Fuzzy *C*-means (FCM) is one of the commonly used algorithms for region-based segmentation of brain tumors. In essence, the classification of each pixel value is achieved through an iterative objective function [3, 4]. Szilágyi et al. [5] proposed a multiple FCM cascade algorithms model, but this model is trained and tested only on a limited data set, with a general degree of generalization; in addition, there is an improved method based on FCM for brain tumor image segmentation [6, 7]. The threshold segmentation algorithm uses image gray value as a similarity measure, which can be categorized into the global threshold and local threshold. The global threshold can be used to make coarse segmentation of the whole tumor area first, so it is often used as the first step in the segmentation process. This method is used to locate the lesion area [8]. If there is a situation where multiple substructures need to be segmented, multiple thresholds can be set for the segmentation of substructures. In addition, threshold segmentation can be combined with multiple segmentation methods to target brain tumor image segmentation. Watershed algorithm (watershed) is a mathematical morphology method [9], which is also widely used in brain tumor image segmentation [10–12]. Although region growth has a wide range of applications in brain tumor segmentation tasks [13–16], the descriptive edge of this method needs to be improved.

With the development of machine learning and deep learning, automatic methods have gradually been applied to the field of brain tumor image segmentation. The emergence of the fully convolutional neural network [17] takes semantic segmentation to an unprecedented step. Many researchers focus their attention on methods using deep learning to achieve fully automatic segmentation of brain tumors through various brain tumor segmentation algorithms. Among them, many machine learning algorithms such as random forest classifiers, clustering, and MRF models are used to solve multimodal MRI brain tumor segmentation problems [18–20]. Recently, in the BraTS competition, we can often see that the segmentation method based on deep learning is proposed. The segmentation method based on the convolutional neural network has the advantage of extracting high-level complex features from the input data, and its excellent feature extraction ability for brain tumor segmentation can be further improved. Deep neural networks have gradually achieved extraordinary results in tasks such as image classification and target detection. Havaei et al. [21] proposed a parallel path CNN model in the field of brain tumor image segmentation to improve the accuracy of brain tumor segmentation; Pereira et al. [22] proposed the use of a convolutional layer with a small-size convolution kernel while reducing the number of network parameters, deepening the number of layers to improve brain tumor segmentation accuracy, and segmentation prediction for malignant tumors and benign tumors; Qamar et al. [23] proposed a neural network structure based on three-dimensional data for brain tumor image segmentation preferably utilized the spatial information of brain tumor images. In addition, many brain tumor segmentation methods based on deep learning methods have been successively proposed [24–28].

Recently, the advancement of medical diagnosis and treatment technology has significantly raised the average life expectancy of brain tumor patients. Moreover, the development of noninvasive imaging methods such as magnetic resonance imaging (MRI) and computer tomography (CT) provides more detailed brain tissue images with a great reference value for the clinical diagnosis of brain tumors and enhances the detection rate. Among various imaging technologies, MRI is the best noninvasive imaging technique, which can detect brain tissue and display three-dimensional images without damaging the healthy tissues. Different MRI pulse sequences can be used to obtain different structure development, and such a set of images is called a multimodal MRI image. MRI images of different modalities have different characterization advantages for the lesion area. Considering from the perspective of a professional physician, at the same time, a comprehensive analysis of MRI images of various modalities can provide a more detailed understanding of the patient's tumor area. Since monomodal MRI images display less information, therefore multimodal MRI images are utilized to accurately segment the lesion area. So currently, professional physicians preferred multimodal MRI images to diagnose the patient's lesion area.

Computer-assisted diagnosis and treatment systems have always been one of the most important topics in medical image processing, especially in the clinical diagnosis and treatment of brain tumors. Different professional doctors will have certain differences in the measurement of tumors. The use of computer-assisted diagnosis and treatment systems can help doctors to measure the exact location and size of the lesion area. So, it becomes more convenient to track and analyze the patient's condition and then specify surgical plans accordingly. To express the significance and practical application of brain tumor segmentation algorithms, Medical Image Computing and Computer-Assisted Intervention Society (MICCAI) conference has held 7 consecutive competitions for brain tumor image segmentation (BraTS). This international conference has greatly promoted the improvement in medical image segmentation technology. Therefore, we propose a cascade network model based on a complete convolution neural network to improve the tumor core region, improve the segmentation accuracy of the tumor region, and obtain good substructure segmentation prediction results on the BraTS 2017 data set.

## 2. Method

### 2.1. Brain Tumor Segmentation Based on Fully Convolutional Neural Network

With the extension of end-to-end training technology, pixel-based image segmentation tasks have achieved unprecedented development. Although conventional neural networks have many problems in the application of image segmentation, which have successfully expanded the application range of convolutional neural networks, fully convolutional neural networks not only have the same advantage of sharing local receptive field weights as convolutional neural networks but also solve convolution. This section mainly describes the fully convolutional neural network model, focusing on the deconvolution method used in the network structure, starting from the brain tumor segmentation problem using multimodal MRI images, and constructing a U-Net network architecture of image segmentation.

#### 2.1.1. Codec Network Model

The fully convolutional neural network structure contains two parts: encoding and decoding. The operation of the convolution process is equivalent to the encoder in the network, that is, the feature extractor, which is extracted from the input data set after a layer of the convolution operation. For the target feature of the image, the operation of increasing the image resolution is equivalent to the decoding part, that is, the feature generator, which is used to increase the resolution of the feature map to calculate the classification result of the pixel, and finally outputs the predicted segmentation map. The application of the fully convolutional neural network model is mainly manifested in unsupervised learning, visual understanding of the network, and research on target generation and semantic segmentation. The biggest difference between the codec network and the convolutional neural network commonly used for classification is the convolution of the fully connected layer and the addition of an operation to increase the resolution of the feature map in the decoding network. The decoding part is mainly composed of a deconvolution layer and a nonlinear activation function layer. The extracted feature map is input into the decoding part of the neural network, and then, the final output is obtained through the nonlinear function activation layer and the deconvolution layer in turn.

#### 2.1.2. Upsampling Module

In pixel-level image segmentation tasks, it is necessary to set up a deconvolution layer in the network structure to improve the resolution of the image. This can be achieved by adopting the following two paths: (1) interpolation method, which belongs to the category of mathematical operations. The more classic ones include bilinear interpolation and cubic difference. To enlarge the size of the input data, it is necessary to fill in the adjacent pixel values in the black pixel area. FCN utilizes bilinear interpolation to perform image upsampling operation, and the value of surrounding pixels is calculated to obtain the value of the intermediate point, to achieve the purpose of increasing the size of the picture. Because of the mathematical operations involved, the parameters are learned without network training. Moreover, the training time can be reduced, and the segmentation efficiency could be improved. (2) Another method is to improve the resolution of the image by transposing the convolution operation, where the learnable convolution layer is consistent with the convolution operation in the ordinary CNN, and both need to undergo the sliding window operation to train the weight coefficients and transpose the volume build-up layer, also known as the deconvolution layer, which can be understood as the inverse process of the convolution operation in form.

#### 2.1.3. Construction of Brain Tumor Image Segmentation Network

The previous article fully discussed the necessity of upsampling in the image segmentation task and elaborated on the main points and objectives of the key layers. Based on the successful application of the U-Net network structure in medical image segmentation tasks, this section constructs a U-Net-based brain tumor segmentation benchmark network structure. The network structure is shown in Figure 1, which will be referred to as a U-Net-based network.

The input data of the segmentation network designed in this section is composed of four modal MRI images (in the order of Flair, T2, T1, and T1C) to form a four-channel image. The specific operation is to use the channel series connection, and then after the convolution operation is executed, the output feature map will be stored, in the decoding part. The output feature map after each layer of upsampling will be a series operation with the previously stored feature map at the corresponding position. The term concatenation operation first appeared in the inception structure in Google Net. Concatenation is the merging of feature maps after convolution operations on different convolution kernels. The feature maps are connected in depth. For example, the input image is a 3 × 3 × 64. Let it be connected in series with the 3 × 3 × 64 feature map; after the series operation, it becomes 128 channels, which is 3 × 3 × 128 output. Through concatenation operation, local information can be fully combined to enrich the information of feature maps. At the same time, the number of feature maps can be halved layer by layer through the convolution layer in the deconvolution module, which greatly reduces memory consumption.

#### 2.1.4. Parallel Dice Loss Structure

In the classification task, the input data is usually classified through the SoftMax layer. For the multimodal MRI brain tumor image segmentation task processed in this paper, four categories need to be output. In medical image processing, the lesion area of interest often only occupies a small area, which is not visible in natural target detection tasks. For the BraTS 2017 data set alone, the number of pixels of the background category label is hundreds of times the number of pixels of the enhanced tumor category label leading to category imbalance in the data. The existence of such a situation directed us toward the process of learning and training. But a local minimum of the loss function is more biased towards background information, leading to the loss of foreground information so that only partial detection results can be achieved. To overcome the problem of imbalanced categories, this paper introduces the Dice loss function to be applied to the brain tumor image segmentation task. The prediction result of using Dice loss will be better than the loss function projected through weighted polynomial logistic regression. The loss function applied to the task of brain tumor image segmentation can be expressed as the following form:

(1) $$\begin{array}{c} L_{dc}=-\frac{2}{\left|K\right|}\underset{K}{\sum }\frac{\sum_{i}p_{ik}g_{ik}}{\sum_{i}p_{ik}+\sum_{i}g_{ik}}. \end{array}$$

Compared with the loss function often used in natural scenes, the Dice loss function introduced in the network can alleviate the problem of imbalance of categories to a certain extent and is more suitable for the brain tissue structure that occupies a smaller area in the task of brain tumor image segmentation. To further improve the accuracy of substructure segmentation, this paper studies a parallel Dice loss scheme. The overall optimization process is shown in Figure 2. Three Dice loss functions are used to calculate the loss of the entire tumor, the tumor core area, and the enhanced tumor area. Theoretically speaking, the parallel Dice loss structure not only balances the segmentation prediction effect of the neural network on the entire tumor but also the enhanced tumor area and the tumor core area. On the other hand, it assigns greater weight to the substructure, which can be segmented and predicted in the result.

### 2.2. Segmentation Based on Cascade Network and Multimodal Images

The previous article elaborated on the feasibility of the application of the fully convolutional neural network in brain tumor image segmentation tasks and constructed a U-Net_based network structure suitable for brain tumor image segmentation. It only needs to extract 2D MRI images through ITK-snap software. The slice data can be used as input data. Using this method can effectively segment the entire lesion area. However, in terms of the nature of MRI images of brain tumors, the edges of substructures are difficult to refine, and the segmentation effect of substructures in brain tumor segmentation tasks is generally poor. To further improve the accuracy of the substructure prediction results, this paper studies the segmentation method based on the U-Net_based network. The first step is to set two categories for segmentation to obtain the prediction of the complete tumor area and return the coordinate information. The next step is to segment the tumor substructure in the tumor prediction area to obtain more accurate substructure segmentation results.

#### 2.2.1. Multimodal MRI Brain Tumor Image Segmentation Framework

Starting from the difficulty of substructure segmentation, this paper studies a cascade network segmentation method based on a U-Net_based network. The cascading network is fabricated by connecting two network structures in series such that the output result of the first network structure is used as the input image of the second network structure. It means that the first network is generally used for training data sets, to get a rough output result; the second network optimizes and improves the accuracy of the output result of the first network. This article sets the use of the first network structure to predict the segmentation results and position coordinate information of the entire tumor, because the network structure can segment the entire tumor more completely, and the second network structure is used to segment the tumor core area and enhanced tumor area. Theoretically speaking, using this kind of network construction method, the problem of multiclass segmentation is transformed into a problem of multiple series-connected segmentation. After extracting the tumor in the entire area in the first network, the second network will segment the substructure based on the first network clipping map, so most of the background information can be clipped. Therefore, the inherent category imbalance of MRI images can be alleviated.

Through this network, characteristic features of each modality in MRI images are properly investigated. In the first stage, the input image uses the serial data of Flair modal and T2 modal images. The fusion of these two modalities can better characterize the entire lesion area. Through network training, the second-class segmentation map of the entire tumor can be obtained. Use the frame to extract it and get the corresponding position information. Then, the extraction results of the entire tumor in the first stage are used as the input of the second stage, and the information of the T1 modal and T1C modal is merged with input data in the second stage for better visualization effect. Since the input image of the second-stage network is smaller than the original image, the multilayer downsampling will lose a certain amount of detailed information, so the number of layers of the network structure is appropriately reduced in the second-stage network. The two network structures in this cascaded network framework use different modal data, which not only enable us to utilize the characteristics information of each modal of multimodal MRI images but also enable us to construct a relatively simple and fully connected network structure under the same conditions. At the same time, the second-stage network reuses the feature maps of the first-stage segmentation prediction, enriching the final segmented feature map information and, overall, enhancing the segmentation of the tumor core area.

#### 2.2.2. Construction of Predicted Network for Substructure Segmentation

To predict the whole area of the tumor, the network structure constructed above with certain amendments is employed. The output category of the model is changed to two categories, to separate the lesion area from the normal tissue area. The novelty of this network structure is that the input image from four serial inputs of two modals is changed to the serial input of the T2 modal and Flair modal image. In addition, the frame extraction operation is added to the network. The input of the training phase includes the truth label and the feature vector, and the frame coordinate information can be output for the second stage of the network.

In the substructure segmentation network, because the input image size will be reduced to a certain extent, consider compressing the number of layers of the network structure, which reduces the convolution module of one unit and the upsampling module of one unit compared with the whole area tumor prediction network. As shown in Figure 3, the network uses four consecutive convolution modules to extract target feature information. Many experiments show that using two small convolution kernels has the same receptive field as using a 5 × 5 convolution kernel, which can reduce the weight parameters and reduce the occurrence of overfitting. The feature extraction stage in the substructure segmentation network continuously uses a 3 × 3 size convolution kernel, and the downsampling layer is set to a size of 2 × 2, which is the same as the whole area positioning network. The downsampling operation is also used to reduce image resolution and reduce network training. The difference between parameters and network settings is that the number of downsampling layers of the convolution part of the substructure segmentation network is reduced to three layers. This situation is usually avoided where the image resolution is greatly reduced, which results in a large loss of image target information.

The input data is an image composed of two modal MRI images (in the order of T1 and T1C) in series. The network also contains two parts of encoding and decoding, and the encoding part is reduced to four convolution modules. The continuous convolution module is used for extracting the target feature information in the input image. The number of feature maps of the first convolution module set in this experiment is 32. From then on, the number of feature maps of each convolution module is doubled until the number of channels increases to 256; in the decoding part, three deconvolutions are set correspondingly to the product module which is used to improve image resolution and dense feature map information. Upsampling operation can choose bilinear interpolation and transposed convolution operation.

## 3. Experiments and Discussions

### 3.1. Evaluation of Upsampling Module

The training comparison of the upsampling module in the U-Net_based network is performed using bilinear interpolation and transposed convolutional layer. As shown in Figure 4, for the convenience of observation, the Dice coefficient variation curve shown in Figure 4 is utilized to observe the effect of the entire area of the tumor. The experimental results shown in Figure 4 predicted that both methods can achieve similar segmentation accuracy. Subsequent experiments in this paper use the bilinear interpolation method for the upsampling process in the network.

### 3.2. Evaluation of Dice Loss

To verify the effectiveness of segmentation, Dice loss is introduced in the brain tumor image segmentation task, and to further test the optimization performance, parallel Dice loss structure is instigated. The quantitative analysis results of the specific prediction results on the test set are shown in Figures 5 and 6. First, it is confirmed that the introduction of the Dice loss function can improve the accuracy of the network prediction results. On the other hand, from the data in the table, it can be known that the parallel Dice loss structure can, to a certain extent, not only improve the accuracy of the network prediction results but also improve the segmentation effect of the tumor core area and the enhanced tumor area.

### 3.3. Comparison with Other Methods

Table 1 summarizes the horizontal comparison results of the parallel Dice loss structure, cascade network, and other methods in this section of the experiment. The measurement data records the average value of multiple experimental results, and the Haus distance index records the 95% percentile value. This paper selects two lateral comparison experiments that are also based on the U-Net network model of the brain tumor segmentation model, which proves the effectiveness of the experiment under the same conditions network structure. Among them, this paper builds the brain network based on the previously available literature [29]. The tumor segmentation network model was trained and tested on the BraTS 2017 data set, and the test results were obtained.

From the quantitative analysis of the prediction results on the test set, the Dice index value is slightly lower than that of the validation set. It is necessary to consider the large differences between different patients. The test results of the test comparison set are not as good as that of the validation set. The index value is high. But no matter which set of experimental data it is, it shows that the segmentation effect of the whole area of the tumor is better, mainly because the area of the whole area of the tumor is relatively large, and the edge gray value of the connection with the normal tissue is different, so it can improve the segmentation of the whole area of the tumor.

Through horizontal comparison, the segmentation algorithm studied in this chapter does not have much advantage in the segmentation effect of the entire tumor, but it can accurately improve substructure segmentation. Among the three evaluation indexes, the Dice coefficient is mainly evaluated as the accuracy criterion. When the Dice index is equal, the Sens and Haus indexes are considered. In the prediction results of core region segmentation, the cascade framework reflects the advantages of segmentation of tumor core regions. The analysis of the segmentation prediction results of the entire tumor and the enhanced tumor region is the same. On the one hand, you can see the effectiveness of the parallel Dice loss structure application; on the other hand, it proves that the use of the cascade network framework greatly improves the tumor core area, enhances the tumor area, and improves segmentation accuracy.

## 4. Conclusions

Multimodal MRI brain tumor image segmentation task, segmenting the entire tumor and tumor core area, enhanced tumor area from normal brain tissue. The research on computer-aided diagnosis and treatment of multimodal MRI brain tumor image segmentation has always been an important topic in the field of medical image processing. The difference in imaging equipment and imaging conditions will cause even the same patient in the same period to have a different MRI with different properties. There are also certain differences in MRI images of brain tumors, and most of the MRI images of brain tumors have obvious bias field strengths, and there are uneven grayscale differences between different patients. In addition, the focus area is different from normal cell tissues. The grayscale similarity between regions is greater, and the edge between the tumor core region and the enhanced tumor region is more complicated. In this context, this paper takes the deep learning method as a tool, makes full use of the complementary feature information between multiple modes, establishes a network model suitable for brain tumor segmentation task based on the full convolution neural network framework, adopts the end-to-end training method, and uses the two-dimensional slice of MRI image as the network input data. Aiming at the imbalance of brain tumor image data categories, the Dice loss function is introduced into the network to calculate the network training loss. At the same time, to further improve the segmentation effect of substructure, a parallel Dice loss structure is studied in this paper. To improve the tumor core region and improve the segmentation accuracy of the tumor region, this paper constructs a cascade network model based on the complete convolution neural network framework and achieves a good prediction effect on the substructure segmentation on the BraTS 2017 data set. However, this study has not been clinically tested, and the clinical accuracy needs to be further explored.

## Figures and Tables

**Figure 1:** The basic framework of U-Net based network.

**Figure 2:** The basic framework of the parallel Dice loss structure.

**Figure 3:** Network framework for substructure segmentation of brain tumor.

**Figure 4:** Comparison of different upsampling methods.

**Figure 5:** Quantitative analysis of Dice loss on Dice.

**Figure 6:** Quantitative analysis of Dice loss on Haus.

**Table 1:** Comparison of test segmentation results.

Region	Method	Dice	Sensitivity	HD
WT	Literature [27]	0.84	0.87	10.3
	Literature [29]	0.88	0.89	8.8
	Ours	0.85	0.86	9.7
TC	Literature [27]	0.72	0.76	16.0
	Literature [29]	0.76	0.74	13.0
	Ours	0.79	0.79	8.6
ET	Literature [27]	0.65	0.65	7.4
	Literature [29]	0.74	0.78	6.5
	Ours	0.75	0.74	4.2

## Data Availability

The data sets used and analyzed during the current study are available from the corresponding author upon reasonable request.
